The article "Intestinal Flora Balance Therapy Based on Probiotic Support Improves Cognitive Function and Symptoms in Patients with Alzheimer's Disease: A Systematic Review and Meta-analysis" was retracted in 2023. Reasons: signs of a paper mill; compromised peer review; unreliable results or conclusions.

# Intestinal Flora Balance Therapy Based on Probiotic Support Improves Cognitive Function and Symptoms in Patients with Alzheimer's Disease: A Systematic Review and Meta-analysis

**DOI:** 10.1155/2022/4806163

**Published:** 2022-08-16

**Authors:** Changxing Liu, Xinyi Guo, Xiang Chang

**Affiliations:** ^1^Shaanxi University of Traditional Chinese Medicine, Xianyang 712046, China; ^2^Xi'an Hospital of Traditional Chinese Medicine, Shaanxi Province 710016, China

## Abstract

**Objective:**

The clinical value of intestinal flora balance therapy based on probiotic support in improving cognitive function and symptoms of patients with Alzheimer's disease was to systematically evaluate, so as to provide evidence-based medicine basis for the promotion and use of this therapy.

**Methods:**

The randomized controlled trials (RCTs) were searched for the improvement of cognitive function and symptoms of patients with Alzheimer's disease by intestinal flora balance therapy supported mainly by probiotics in PubMed, EMBASE, ScienceDirect, Cochrane Library, China Knowledge Network Database (CNKI), China VIP database, Wanfang database, and China Biomedical Literature Database (CBM) online database (RCT). Data were extracted independently by two researchers, and the literature was assessed for risk of bias according to the Cochrane Handbook 5.1.0 criteria. The data were meta-analyzed using RevMan 5.4 statistical software.

**Results:**

Finally, 5 randomized controlled trials were included, with a total sample size of 386 cases. The results of meta-analysis showed that Chi^2^ = 13.14, df = 2, *P* = 0.001, and *I*^2^ = 85% showed significant heterogeneity in the inclusion of the study data. Probiotic-supported intestinal microflora balance therapy improves cognitive function in patients with Alzheimer's disease. Through meta-analysis of transient memory scores, it is concluded that intestinal flora balance therapy based on probiotic support can improve transient memory in patients with Alzheimer's disease. Meta-analysis of ADAS-COG score showed that intestinal flora balance therapy supported by probiotics could improve the cognitive function of patients with Alzheimer's disease. The ADL score was analyzed by meta, and the heterogeneity test result was Chi^2^ = 0.79, df = 1, *P* = 0.37 > 0.05, and *I*^2^ = 0%, indicating that the intestinal flora balance therapy supported by probiotics can improve the ability of daily living of patients with Alzheimer's disease.

**Conclusion:**

Intestinal flora balance therapy based on probiotic support can effectively improve cognitive function, instantaneous memory, and ability of daily life in patients with Alzheimer's disease. However, more studies and long-term follow-up studies with higher methodological quality are needed to further verify.

The article "Intestinal Flora Balance Therapy Based on Probiotic Support Improves Cognitive Function and Symptoms in Patients with Alzheimer's Disease: A Systematic Review and Meta-analysis" was retracted in 2023. Reasons: signs of a paper mill; compromised peer review; unreliable results or conclusions.

## 1. Introduction

In recent years, with the extension of human life, the problem of aging population is becoming more and more serious. The quality of life of the middle-aged and elderly will be affected by many factors, especially various chronic diseases. Among the chronic diseases of the elderly, neurological diseases are more common and serious, including stroke, Alzheimer's disease, and Parkinson's syndrome [1]. Alzheimer's disease (AD) is a degenerative disease of the central nervous system that mostly occurs in the elderly or presenile. It is manifested as a progressive decline in cognitive and memory function and ability of daily living, accompanied by a variety of neuropsychiatric symptoms and behavioral disorders [2]. It is the dementia disease with the most extensive influence and the largest number of patients in the world [3]. According to the International Association for Dementia, there are currently more than 55 million people suffering from dementia worldwide. The total number of cases is expected to reach 152 million in 2050 with an average of one disease every three seconds [4]. According to statistics, China has more than 10 million AD patients, ranking first in the world. Moreover, our country is also one of the countries with the fastest growth in the number of patients [5]. With the rapid growth of the elderly population and the increase of human life expectancy year by year, the incidence of AD will increase greatly, seriously endangering the physical and mental health of the elderly. The main pathological features of AD include massive loss of cholinergic neurons and their synapses in cerebral cortex and hippocampus, vascular amyloidosis in cortical arteries and arterioles, accumulation of amyloid *β*-amyloid protein (A*β*), and abnormal hyperphosphorylation of tau protein to form neurofibrillary tangles [6]. According to AD's theory of inflammation, AD may be a chronic inflammatory response of the central nervous system. There is A*β* accumulation in the hippocampus and cerebral cortex of patients with AD. At the same time, glial cells in brain tissue are abnormally activated and secrete a variety of inflammatory substances, resulting in neuronal death and the loss of neural function, finally the occurrence of AD [7].

In recent research findings, there is a certain relationship between brain microbial infection and the occurrence of AD [8]. For example, in specific susceptible people, such as individuals carrying apolipoprotein E-*ε* 4 (APOE-*ε* 4) allele, the blood-brain barrier permeability changes; pathogens such as herpes simplex virus type 1 (HSV-1) can invade the brain and cause chronic inflammation in the brain, which may be related to the occurrence of AD [9]. A large number of studies have shown that intestinal flora plays an important role in regulating intestinal-brain function [10]. The sympathetic and parasympathetic branches of the autonomic nervous system can affect the circuit of the intestinal nervous system and lead to changes in intestinal motility, thus affecting the entry of nutrients from probiotics such as resistant starch, dietary fiber, or other key intestinal microorganisms into the small intestine and colon, thus affecting the balance of intestinal microecology [11]. In addition, the hypothalamic-pituitary-adrenal (HPA) axis can affect the colonization and composition of intestinal flora by stimulating the secretion of adrenocortical hormones [12]. In turn, gut microbes and their metabolites can mediate neurophysiological processes including neurodevelopment, neurotransmission, immune activation of the central nervous system, and the integrity of the blood-brain barrier by regulating the maturation of microglia and astrocytes [13]. In the meanwhile, intestinal flora and their metabolites, such as short-chain fatty acids (SCFAs), *γ*-aminobutyric acid (GABA), and brain-derived neurotrophic factor (BDNF), have important effects on nerve inflammation, nerve injury, and brain behavior by regulating peripheral immune response [14]. Therefore, the composition and function of intestinal microorganisms is a new way to improve nervous system diseases and develop corresponding prevention and treatment methods.

The article "Intestinal Flora Balance Therapy Based on Probiotic Support Improves Cognitive Function and Symptoms in Patients with Alzheimer's Disease: A Systematic Review and Meta-analysis" was retracted in 2023. Reasons: signs of a paper mill; compromised peer review; unreliable results or conclusions.

Probiotics are a large group of live microorganisms that are beneficial to the human body, including lactic acid bacteria and bifidobacteria, which can play the role of probiotics by regulating the intestinal microecological balance. A number of studies have shown that the intake of certain probiotics can effectively prevent and improve AD through the gut-brain axis. The potential mechanisms include regulating intestinal microecology, regulating the metabolism of key substances such as tryptophan, promoting the release of neurotransmitters and other beneficial metabolites, and reducing intestinal permeability and inflammation [15, 16]. Based on this, meta-analysis was carried out by evaluating the clinical value of intestinal flora balance therapy supported by probiotics in improving cognitive function and symptoms in patients with Alzheimer's disease in this study.

## 2. Research Contents and Methods

### 2.1. The Sources and Retrieval Methods of Documents

According to the principles of PICOS (research object, intervention, comparison, outcome, and research design), the retrieval strategy was formulated. Search the Chinese Academic Journal full-text database (CNKI), Wanfang database (Wanfang data), China Biomedical Literature Database (CBM), PubMed, and Web of Science (SCI) database from the establishment of the database to March 2022 which published the clinical research literature of probiotics in the treatment of Alzheimer's disease. Key words such as “probiotics”, “intestinal flora”, “Alzheimer's disease”, and “Alzheimer's disease” were used to search the keywords in the Chinese database. At the same time, the search scope of the retrieved literature was expanded by consulting its references. The literatures containing “random” and “grouping” can be regarded as RCT.

The article "Intestinal Flora Balance Therapy Based on Probiotic Support Improves Cognitive Function and Symptoms in Patients with Alzheimer's Disease: A Systematic Review and Meta-analysis" was retracted in 2023. Reasons: signs of a paper mill; compromised peer review; unreliable results or conclusions.

### 2.2. Literature Inclusion Criteria and Exclusion Criteria

#### 2.2.1. Literature Inclusion Criteria

(1) Study type: RCT of intestinal flora balance therapy based on probiotic support in the treatment of AD, whether blind or not. (2) Subjects: adopt accepted and clear diagnostic criteria for AD. The patient's age, gender, and case source are not limited. (3) Intervention: the observation group was treated with probiotics or combined with other drugs, and the control group was treated with nonprobiotics.

#### 2.2.2. Literature Exclusion Standard

(1) It was not a randomized controlled study. (2) The data report was incomplete, and the data cannot be used. (3) It was a repetitive research. (4) The diagnostic criteria and curative effect evaluation were not clear. (5) The subjects in the trial did not rule out other diseases causing cognitive impairment (such as cerebrovascular diseases).

### 2.3. Quality Evaluation and Data Extraction

#### 2.3.1. Quality Evaluation

Referring to the systematic evaluation manual of Cochrane intervention measures (version 6.1), the risk bias assessment tool of the RevMan 5.4 software was used for quality evaluation. Two researchers independently assessed risk of bias for included RCTs. If conclusions were inconsistent, discrepancies were resolved by discussion or by introducing the judgment of a third researcher

#### 2.3.2. Data Extraction

Two evaluators independently extracted and cross-checked the literature. When the two people had differences, they reached an agreement through consultation. It included the study author, publication time, sample size, treatment method, curative effect evaluation method, and so on.

### 2.4. Statistical Processing

The RevMan 5 software originated from Cochrane collaboration network for meta-analysis. The mean and standard deviation of the net change difference of serum albumin, prealbumin, and hemoglobin in the experiment and the control cohorts were input into RevMan 5 for analysis. Because the index is a continuous variable, the weighted mean difference (WMD) is used as the effect scale, and 95% confidence interval is selected. First, *X*^2^ test is used to determine whether there is heterogeneity between the studies; if *P* > 0.05 and *I*^2^ < 50%, it is considered that the included study is homogeneous, and the modified impact model can be collected for meta-analysis. If *P* < 0.05 and *I*^2^ ≥ 50%, when judging the homogeneity of the included study, the combined effect is needed; then, choose the random effect model. If *P* < 0.05 and the source of heterogeneity could not be judged, meta-analysis was not performed, and descriptive analysis was used.

The article "Intestinal Flora Balance Therapy Based on Probiotic Support Improves Cognitive Function and Symptoms in Patients with Alzheimer's Disease: A Systematic Review and Meta-analysis" was retracted in 2023. Reasons: signs of a paper mill; compromised peer review; unreliable results or conclusions.

## 3. Results and Analysis

### 3.1. The Results of Literature Retrieval and the Basic Situation of Literature Inclusion

2211 articles were retrieved by computer database, 466 articles were obtained after eliminating repeated studies, 67 articles were obtained by preliminary reading of the titles and abstracts, and 15 articles were included after excluding irrelevant studies, reviews, case reports, and noncontrol literatures. Then, 10 articles with incomplete data and no main outcome indicators were read carefully, and in the end, 5 RCTs were enrolled [17–21]. Totally, 386 samples were analyzed by meta. The basic features of the included literatures are shown in Table 1.

### 3.2. Evaluation of the Quality of the Methodology Included in the Literature

The five RCT literatures are included in this investigation. All reported the baseline of patients, and 4 RCTs mentioned “random allocation.” However, the allocation method is not specified. Detailed interventions and follow-up times were given for the five included studies. 5 RCT articles did not describe in detail the number and reasons for blinding and loss to follow-up or dropout. The literature risk of bias is shown in Figures 1 and 2.

### 3.3. Meta-analysis Result

#### 3.3.1. MMSE Scoring

Through the inclusion of 5 RCT studies, the MMSE scores between the research group and the control group were analyzed by meta. The heterogeneity test results displayed the great heterogeneity among the included data (Chi^2^ = 13.14, df = 2, *P* = 0.001, *I*^2^ = 85%). This showed that there was a significant heterogeneity among the included data. It considered that intestinal flora balance therapy based on probiotic support can improve the cognitive function of patients with Alzheimer's disease. All the results are shown in Figure 3.

#### 3.3.2. Instant Memory Score

Through the meta-analysis of the instantaneous memory scores of 386 samples involved in the two groups in 5 RCT studies, the results of heterogeneity test exhibited the heterogeneity among the included data by Chi^2^ = 15.11, df = 1, *P* = 0.0001, and *I*^2^ = 93%. Through the analysis of Figure 4, it suggested that intestinal flora balance therapy based on probiotic support can improve the instantaneous memory of patients with Alzheimer's disease.

The article "Intestinal Flora Balance Therapy Based on Probiotic Support Improves Cognitive Function and Symptoms in Patients with Alzheimer's Disease: A Systematic Review and Meta-analysis" was retracted in 2023. Reasons: signs of a paper mill; compromised peer review; unreliable results or conclusions.

#### 3.3.3. ADAS-cog Scoring

Through the meta-analysis of the ADAS-cog scores in the research group and the control group, the heterogeneity test results showed Chi^2^ = 27.12, df = 2, *P* < 0.00001, and *I*^2^ = 93%, indicating that there was obvious heterogeneity among the included research data. This suggested that probiotic-supported gut microbiota balance therapy may improve cognitive function in Alzheimer's disease patients (Figure 5).

#### 3.3.4. ADL Scoring

Through the meta-analysis of ADL scores of 386 samples involved in the research group and the control group, the heterogeneity test results were Chi^2^ = 0.79, df = 1, *P* = 0.37, and *I*^2^ = 0%, indicating an obvious heterogeneity among the included research data. Additionally, the combined effect WMD was analyzed by random effect model. From the analysis in Figure 6, it could be seen that the combined effect size WMD test was *Z* = 15.31 (*P* < 0.00001). According to the analysis results, it could be concluded that the use of probiotic support-based intestinal flora balance therapy was effective for Alzheimer's disease. The patient's ability of daily living had been improved.

## 4. Discussion

AD is one of the most common diseases in the elderly, and the incidence of AD is increasing year by year with the aging of the population. AD is mainly manifested by progressive cognitive impairment, abnormal mental behavior, and decreased ability of daily living, which is the most common type of senile dementia [22]. The pathological features of AD are extracellular senile plaques formed by the deposition of amyloid *β*-amyloid (A*β*) and intracellular neurofibrillary tangles formed by hyperphosphorylation of tau protein, as well as neuronal loss with gliosis [23]. No consensus has been reached on the pathogenesis of AD. Previous studies have suggested that the pathogenesis of AD is related to the imbalance of intestinal flora. The imbalance of intestinal flora will lead to the disorder of “microorganism-intestinal-brain axis.” Too much metabolite ammonia enters the blood circulation, which will affect the central nervous system and may be involved in the pathogenesis of AD [17, 24]. Previous studies have found the alterations in the composition of gut microbes affect the permeability of the gut wall. A large number of neurotransmitters in the gut can ascend to the central nervous system via the “microbe-gut-brain axis,” and the metabolites of bacteria in the gut can lead to neuroinflammation [21, 22]. There are various microorganisms in various parts of the human body, such as the skin, mouth, and intestines. The intestine is the area where the largest microflora is located in the human body, including bacteria, archaea, viruses, and eukaryotes. Most of them are bacteria, about 100 trillion involving more than 1,000 species, which is 10 times the number of cells in our whole body and 150 times the number of human genomes [22–24]. Gut microbes play a very important role in maintaining human health. They can promote the digestion and absorption of nutrients, resist the invasion of foreign bacteria, regulate the body's immunity, and participate in the metabolic processes of the human body and the biosynthesis of vitamins. Firmicutes and Bacteroidetes account for the majority of gut microbes, while Actinobacteria, Proteobacteria, Fusobacterium, Verrucobacterium, and Cyanobacteria account for a small number [25]. The differences in the number, proportion, and abundance of spores correlate with the health of the host. The intestinal flora and the host are interdependent and restricted to maintain a dynamic balance. A balanced intestinal flora can promote the health of the host. When the external environment changes or the host's own factors change, it can cause intestinal flora imbalance, damage to the intestinal mucosal barrier and decline in the body's immunity, and induce various diseases. There is bidirectional regulation between the gastrointestinal tract and the central nervous system, and this interacting pathway is called the “microbe-gut-brain axis” [26]. The “microbe-gut-brain axis” includes the digestive tract, gut microbes, enteric nervous system, autonomic nervous system, and central nervous system. The gut and brain mainly interact through a variety of complex mechanisms such as the nervous system, the endocrine system, and the immune system. From bottom to top, the autonomic nervous system transmits information from the intestinal lumen to the central nervous system through enteric, spinal, and vagal pathways [27]. The central nervous system also regulates effector cells in the gastrointestinal tract through the autonomic nervous system. Neuroendocrine pathways are regulated through the “hypothalamic-pituitary-adrenal axis.” Immune regulation is accomplished by the intestinal immune system formed by immune cells in the intestinal mucosa and secreted immunoglobulin A. The gut microbiota influences neurodevelopment, cognition, and behavior through these pathways [28].

The article "Intestinal Flora Balance Therapy Based on Probiotic Support Improves Cognitive Function and Symptoms in Patients with Alzheimer's Disease: A Systematic Review and Meta-analysis" was retracted in 2023. Reasons: signs of a paper mill; compromised peer review; unreliable results or conclusions.

Comparing with the fecal flora and blood inflammatory factors between AD and non-AD patients, the abundance of rectal true bacilli with anti-inflammatory effect in the fecal flora of AD patients decreased. The abundance of Shigella proinflammatory increased, which was positively correlated with the level of inflammatory factors and the severity of AD [29]. The change of flora diversity may trigger neuroinflammation, A*β* aggregation, and tau protein pathological changes. In the process of human aging, the alterations of AD-like were also found, and intestinal probiotics decreased, and proinflammatory bacteria increased [30]. The composition of intestinal flora in patients with AD is basically consistent with the physiological succession of human intestinal flora, which may prove why AD is an age-related disease and is prone to high incidence in the elderly. It is generally believed that the intestinal tract of the fetus is aseptic and the intestinal bacteria of the newborn comes from a large number of microbes that come into contact with the mother and the environment during childbirth. These microorganisms are highly variable in infancy and gradually stabilize in childhood. Finally, they are colonized in the gastrointestinal tract, similar to the composition of microorganisms in adults. With the increase of age, the diversity of intestinal microorganisms gradually will change; the number of beneficial bacteria will decrease. As a living functional microorganism, the efficacy of probiotics against AD has been gradually developed, including in vitro index detection, animal model analysis, and clinical trials [31]. In recent years, some studies have found that the diversity of intestinal flora in patients with AD decreased significantly, the species and abundance of intestinal flora changed, the abundance of Bacteroides increased, and the abundance of thick-walled bacteria and bacilli decreased [32]. Cronin et al. [33] found that the more severe the cognitive impairment of AD patients, the lower the diversity of the gut flora. Thus, the degree of cognitive impairment in AD patients may be related to specific flora. Many animal experiments have also verified the correlation between the changes of intestinal flora and AD. Chang et al. [34, 35] sequenced the bacteria in the feces of amyloid precursor protein transgenic mice by 16SrRNA and found that the intestinal microflora changed significantly compared with nontransgenic wild-type mice. The levels of Streptomyces, Proteus, actinomycetes, and verrucous microorganisms in intestinal microorganisms decreased, while the levels of Bacteroides and soft-walled bacteria increased. Changes in gut microbial composition affect the maturation and function of the gut mucus layer, leading to disruption of the gut barrier. After increased intestinal permeability, harmful substances enter the immune system, which in turn disrupts the blood-brain barrier, leading to neuroinflammation. Intestinal microorganisms can produce neurotransmitter precursors or neurotransmitter uplink to regulate central nervous function, affecting learning, memory, and cognitive function. The central nervous system can also produce neurotransmitters or hormones descending to affect the composition of intestinal microorganisms. The total level of neurotransmitters in the intestinal tract may be higher than that in the brain, and the neurotransmitters in the intestinal tract can regulate intestinal motility, intestinal cell secretion, and signal transduction. These neurotransmitters include *γ*-aminobutyric acid (GABA), serotonin, dopamine, and norepinephrine [36]. GABA is the main inhibitory neurotransmitter in the central nervous system, a nonprotein amino acid produced by L-glutamate under the action of glutamate decarboxylase. Bacteria in the intestinal tract, especially Lactobacillus and Bifidobacterium, can produce GABA, activate sensory signals in the gastrointestinal wall, and regulate the central nervous system through the vagus nerve. GABA entering the bloodstream regulates hormone secretion in the hypothalamus by affecting the hypothalamic-pituitary-adrenal axis. The autopsy of patients with AD found that the level of GABA in parietal lobe, temporal lobe, and frontal cortex decreased, indicating the correlation between AD and GABA deficiency [29], but the specific mechanism needs further study. Thal et al. explored the neuroprotective and behavioral protective effects of Bacillus subtilis NCIB3610 on transgenic AD nematodes [37]. It was found that the strain could significantly alleviate the paralysis phenotype associated with AD and restore the life span of nematodes. The ability of quorum sensing peptide synthesis and intestinal biofilm formation may be the key for Bacillus subtilis to play an anti-AD probiotic effect. A few studies have shown that high intake of probiotics and probiotics can improve neurocognitive ability and reduce the risk of AD disease. In another study, the researchers analyzed the neuroprotective effects of three different probiotics, Lactobacillus plantarum DR7, Lactobacillus DR9, and Lactobacillus casei on transgenic AD Drosophila melanogaster. Lactobacillus plantarum DR7 was the most effective in improving the rough phenotype of AD Drosophila eyes. 16SrRNA sequencing showed that Lactobacillus plantarum DR7 could significantly reduce the abundance of Wolbachia and increase the abundance of Stenotrophomonas and Acetobacter in the intestinal flora of Drosophila melanogaster. Therefore, the authors speculated that Stenotrophomonas and Acetobacter were negatively correlated with AD, and Wolbachia may be a potential target of neurodegenerative diseases such as AD and PD [38]. This study has been the first to link Wolbachia with neurological diseases, which can help people prevent and treat neurological diseases by inhibiting harmful bacteria in the gut. The foreign scholars ever reported that the number of neuronal apoptosis in the brain was reduced after feeding AD animals with oligofructose; the phosphorylation of tau protein was reduced, and the expression of A*β*42 was downregulated. The total 60 AD patients were blindly selected and randomly divided into two groups. They were treated with milk (control group) and probiotics (treatment group) for 12 weeks after treatment, the MMSE score of the treatment group improved [39]. Moreover, the use of Lactobacillus and Bifidobacterium can reduce A*β* deposition in the brain of rats injected with A*β*42 in the hippocampus, promote superoxide dismutase (SOD) production, and reduce serum malondialdehyde (MAD) levels, so Lactobacillus and Bifidobacterium Bacillus can improve AD memory, learning deficits and oxidative stress [40]. Prebiotics and probiotics can delay the progression of AD to a certain extent, showing their potential to treat AD. The cost of this treatment may be relatively cheap, and there are no adverse reactions. It may be used in combination with clinical AD drugs to play a synergy therapeutic effect.

The article "Intestinal Flora Balance Therapy Based on Probiotic Support Improves Cognitive Function and Symptoms in Patients with Alzheimer's Disease: A Systematic Review and Meta-analysis" was retracted in 2023. Reasons: signs of a paper mill; compromised peer review; unreliable results or conclusions.

At present, there is still a lack of high-level evidence-based evidence about the clinical value of intestinal flora balance therapy with probiotic support in improving cognitive function and symptoms in patients with Alzheimer's disease. This paper systematically evaluates the clinical value of probiotic-supported intestinal flora balance therapy in improving cognitive function and symptoms of patients with Alzheimer's disease and provides evidence-based medicine basis for the promotion and use of this therapy. In this paper, 5 randomized controlled trials were included, with a total sample size of 386 cases. The results of meta-analysis showed that Chi^2^ = 13.14, df = 2, *P* = 0.001, and *I*^2^ = 85% showed significant heterogeneity in the inclusion of the study data. Probiotic-supported intestinal microflora balance therapy improves cognitive function in patients with Alzheimer's disease. Through meta-analysis of transient memory scores, it is concluded that intestinal flora balance therapy based on probiotic support can improve transient memory in patients with Alzheimer's disease. Meta-analysis of ADAS-COG score showed that intestinal flora balance therapy supported by probiotics could improve the cognitive function of patients with Alzheimer's disease. The ADL score was analyzed by meta, and the heterogeneity test result was Chi^2^ = 0.79, df = 1, *P* = 0.37 > 0.05, and *I*^2^ = 0%, indicating that the intestinal flora balance therapy supported by probiotics can improve the ability of daily living of patients with Alzheimer's disease. Based on the results of this analysis, it can be considered that the use of probiotic support-based intestinal flora balance therapy can improve the daily living ability of patients with Alzheimer's disease. There are some limitations in this study. First of all, the sample size of the references included in this study is small, and they all belong to single-center research; there is a certain deviation. In the future research, we will carry out a large sample of prospective studies and hopefully draw more valuable conclusions.

The article "Intestinal Flora Balance Therapy Based on Probiotic Support Improves Cognitive Function and Symptoms in Patients with Alzheimer's Disease: A Systematic Review and Meta-analysis" was retracted in 2023. Reasons: signs of a paper mill; compromised peer review; unreliable results or conclusions.

## 5. Conclusion

Probiotic-supported gut microbiota balance therapy can effectively improve cognitive function, transient memory, and daily living abilities in Alzheimer's disease patients. However, more studies and follow-up studies with higher methodological quality and longer intervention time are needed for further verification.

## Figures and Tables

**Figure 1:** Risk of bias chart.

**Figure 2:** Risk of bias summary chart.

**Figure 3:** Forest plot of meta-analysis of MMSE score between the two groups.

**Figure 4:** Forest plot of meta-analysis of instantaneous memory score between the two groups.

**Figure 5:** Forest plot of meta-analysis of ADAS-cog score between the two groups.

**Figure 6:** Forest plot of meta-analysis of ADL score between the two groups.

**Table 1:** Basic characteristics of literature.

Include the literature	Year of publication	*N* (C/T)	Intervention method		Experimental time	Random or not	Blind or not	Outcome index
			Control group	Research group				
Li Xianqiang	2015	14/14	Simo decoction is taken orally	Simo decoction combined with Clostridium butyricum powder	12 months	Yes	No	①
Wang Xiaodong	2014	14/14	Simo decoction is taken orally	Simo decoction combined with Clostridium butyricum powder	12 months	Yes	No	①②
Wang Yunxia	2021	100/100	Routine treatment	Oral Silankang	8 weeks	Yes	No	①③④
Zhu Manlian	2021	35/35	Donepezil	Donepezil + Clostridium butyricum live bacteria capsule	8 weeks	Yes	No	②③④
Ma li	2021	30/30	Galantamine tablets combined with placebo	Galantamine tablets combined with intestinal probiotics	16 weeks	Yes	No	③

① MMSE scoring; ② instant memory score; ③ ADAS-cog; ④ ADL.

## Data Availability

The datasets used and analyzed during the current study are available from the corresponding author upon reasonable request.
